The article "Intravoxel Incoherent Motion Diffusion-Weighted Imaging and 3D-ASL to Assess the Value of Ki-67 Labeling Index and Grade in Glioma" was retracted in 2023. Reasons: signs of a paper mill; compromised peer review; unreliable results or conclusions.

# Intravoxel Incoherent Motion Diffusion-Weighted Imaging and 3D-ASL to Assess the Value of Ki-67 Labeling Index and Grade in Glioma

**DOI:** 10.1155/2022/8429659

**Published:** 2022-08-31

**Authors:** Jian Zhou, Huafeng Li, Xiaoming Ma, Miao Jin, Xin Meng, Guangfeng Zhang

**Affiliations:** ^1^Department of MRI, The Third Affiliated Hospital of Qiqihar Medical University, Qiqihar, Heilongjiang 161000, China; ^2^Department of Endocrinology (I), The Third Affiliated Hospital of Qiqihar Medical University, Qiqihar, Heilongjiang 161000, China; ^3^Department of Ultrasound, The Third Affiliated Hospital of Qiqihar Medical University, Qiqihar, Heilongjiang 161000, China

## Abstract

**Objective:**

To determine the proportion of intravoxel incoherent motion diffusion-weighted images (IVIM-DWI) and three-dimensional arterial circulation markers (3D-ASL) in Ki-67 labeling index (Ki-67 LI) and glioma grading.

**Methods:**

According to the classification of diseases of the central nervous system dealt with by WHO in 2007, patients with stage II glioma were classified as low (*n* = 20) and patients with stages III-IV were divided into higher levels (*n* = 22). Prior to surgery, brain MRI, IVIM-DWI, and 3D-ASL were performed in all patients, and the actual water molecular diffusion coefficient (*D*), microcirculation coefficient (*D*∗), blood flow fraction (*f*), and cerebral blood flow (CBF) were measured. A rank sum (Mann–Whitney *U* test) was used to compare the four upper and lower level Ki-67 LI measurements. Spearman's method is used to identify the relationship between 4 groups of quantification and Ki-67 LI. Reciprocal grafting (ROC) curves were used to measure the diagnosis of four groups of glioma grading defects.

**Results:**

There were significant differences in *D*, *D*∗, *f*, and CBF between the solid region of the tumor and the normal white matter contralateral to it (*P* < 0.05). The significant differences of *rD*, *rD*∗, *rf*, and *r*CBF were shown between patients with low-grade glioma and high-grade glioma (*P* < 0.05). Ki-67 LI was found to have negative correlation with *rD* (*r* = 00.693, *P* < 0.001) and *rf* (*r* = 00.539, *P* < 0.001), but similarly correlated with *r*CBF (*r* = 0.665, *P* < 0.001) in patients with glioma. Recipient efficacy for predicting advanced and secondary glioma from *rD*, *rf*, *rD*∗, *r*CBF, and Ki-67 LI raises AUCs of 0.819, 0.747, 0.719, 0.836, and 0.907, respectively.

**Conclusion:**

IVIM-DWI has good application value for preoperative grading of glioma.

## 1. Introduction

Gliomas are tumors of the brain and are the most common type of cancer in young people, accounting for more than 70% of intracranial cancers [1]. Depending on the stage of leukemia, glioma is divided into stages I-IV. Type I includes pilocytic astrocytoma, pleomorphic xanthoastrocytoma, subependymal giant cell astrocytoma, type II oligodendroglioma, and astrocytoma. High-grade glioma is grade III and is represented by anaplastic oligodendroglioma, anaplastic astrocytoma, anaplastic oligoastrocytoma, anaplastic ependymoma, and grade IV glioblastoma [2]. The incidence rate of glioma is related to a series of factors, including histological type, age, gender, race, and country. It was reported that according to the standardized age, around 4.7 of 100,000 people suffered from glioma every year [3]. The annual age-adjusted incidence of grade IV glioblastoma ranged from 0.59 to 3.69 per 100,000 people, leading to high molarity [4].

The article "Intravoxel Incoherent Motion Diffusion-Weighted Imaging and 3D-ASL to Assess the Value of Ki-67 Labeling Index and Grade in Glioma" was retracted in 2023. Reasons: signs of a paper mill; compromised peer review; unreliable results or conclusions.

In most cases, surgical resection is an important treatment for glioma. It contributed to reduced intracranial pressure, relief of neurological symptoms, and prolongation of overall survival of the patients [5]. Accurate scoring of glioma before surgery is important in clinical selection and prognosis. Magnetic resonance imaging (MRI) procedures are often limited in their sensitivity to neurological changes. Diffusion-weighted magnetic resonance imaging (DWI), which dates back to 1985, has been successfully used to treat neurological disorders, particularly stroke [6]. Intravoxel incoherent motion (IVIM) is a method of seeing water in the 1988 study, which describes the movement of tissue through molecular diffusion and blood microcirculation, which affects the measurement of vision using the apparent diffusion coefficient (ADC) [7]. IVIM scores are critical for survival in glioma patients [8], as well as hyperacute brain stroke [9]. Arterial spin labeling (ASL) is a magnetic resonance perfusion assessment method based on water in the blood as an internal source to quantify the value of cerebral blood flow (CBF) [10]. This assessment method has been widely used in clinical area such as brain tumors [11] and cerebrovascular diseases [12]. The occurrence of glioma has proved to be associated with immune function disorder. Proliferative cancers can be diagnosed by Ki-67 immunohistochemistry, and the Ki-67 labeling index (Ki-67 LI) is widely used in cancer screening [13].

The method of IVIM and ASL is a noninvasive MRI technique without the use of contrast agents and has been applied to the study of glioma, but their diagnostic value remains unclear. So far, rare studies have found correlations between their parameters and Ki-67 LI and glioma score. The purpose of this study was to explore the correlation between IVIM-DWI and 3D-ASL quantitative parameters and Ki-67 LI of glioma and their value in glioma grading evaluation.

The article "Intravoxel Incoherent Motion Diffusion-Weighted Imaging and 3D-ASL to Assess the Value of Ki-67 Labeling Index and Grade in Glioma" was retracted in 2023. Reasons: signs of a paper mill; compromised peer review; unreliable results or conclusions.

## 2. Materials and Methods

### 2.1. Study Design

42 patients with glioma were included in the study between December 2016 and May 2019 at the Third Affiliated Hospital of Qiqihar Medical University. Patient's age ranged from 25 to 83 years, with average 53 ± 12 years. None received radiotherapy, chemotherapy, or steroid therapy prior to MRI examination. Each patient provided complete imaging data and underwent surgical resection within two weeks after MRI examination. Out of 42 patients, 20 patients with grade II, 12 patients with grade III, and 10 patients with grade IV were registered in 2007. The WHO modified the distribution of tumors in the central nervous system and the brain [14], and the classification was confirmed by their films read by two experienced pathologists. Patients with stage II glioma were included in the lower group, and patients with stages III-IV were included in the upper group. Written consent will be obtained from each patient. The curriculum is approved by the Legal Committee of the Third Affiliated Hospital of Qiqihar Medical University. This survey included 42 patients diagnosed with glioma.

### 2.2. Image Acquisition

Hom MR scan: cross-sectional fluid attenuation inversion recovery (FLAIR) sequence T1WI: TR 1850 ms, TE 24 ms, and TI 780 ms; fast spin echo (FSE) sequence T2WI: TR 6656 ms, TE 105 ms, field of view (FOV) 240 mm × 240 mm, matrix 352 × 256, slice thickness 5 mm, interslice spacing 0, and 34 scan layers.

IVIM-DWI: spin-echo single-shot echo-planar imaging (SS-EPI) DWI: TR 4500 ms; TE minimum value; set 13 *b* values of 0, 10, 20, 30, 50, 100, 150, 200, 400, 800, 1200, 2000, and 3000 s/mm^2^; take 2, 1, 1, 1, 1, 1, 2, 2, 3, 3, 5, and 6 as the corresponding excitation times (NEX); and the scanning time is 378 s. FOV 240 mm × 240 mm, matrix 160 × 160, layer thickness 5 mm, interlayer distance 0, and 34 scanning layer.

3D-ASL: FSE-based 3D spiral acquisition with combination of pulse and continuous manners: TR 4594.0 ms, TE 10.1 ms, points 512, arms 8, marking delay time 1525 ms, FOV 240 mm × 240 mm, layer thickness 4.0 mm, no interval, and 24 scanning layers.

Enhanced MR scan: cross-sectional T1WI-enhanced scan: TR 1850 ms, TE 24 ms, TI 780 ms, FOV 240 mm × 240 mm, matrix 352 × 256, slice thickness 0, slice spacing 0, and 34 scan layers.

### 2.3. Image Analysis

The images were transferred to the GE AW 4.5 Image Workstation (USA). The Functool MADC software was used to analyze IVIM-DWI, and 3D-ASL software was used to analyze and to obtain pseudocolor maps. Two neuroradiologists used different models to describe the region of interest (ROI) along the largest inner edge 3D-ASL uptake area of the tumor and then obtained CBF values on tumor and contralateral white matter using MR imaging at the cutoff cyst formation. An ROI (approximately 50 mm^2^) was manually placed in the white matter area opposite the hemorrhagic or necrotic area in the same layer. Based on the ROI of the ASL image, the ROI of the IVIM-DWI image was defined, and the real molecular diffusion coefficient (*D*), microcirculation coefficient (*D*∗), and vacuum (*f*) were doubled in exponential fashion. The ROI size and position of ASL and IVIM-DWI are consistent. Normal contralateral white matter was used for normalization. To obtain the correct molecular diffusion coefficient, the tumor volume was divided by the volume of the contralateral normal white matter (*rD*), relative microcirculation perfusion coefficient (*rD*∗), relative perfusion fraction (*rf*), and relative cerebral blood flow (*r*CBF), so as to avoid individual differences between samples.

The article "Intravoxel Incoherent Motion Diffusion-Weighted Imaging and 3D-ASL to Assess the Value of Ki-67 Labeling Index and Grade in Glioma" was retracted in 2023. Reasons: signs of a paper mill; compromised peer review; unreliable results or conclusions.

### 2.4. Ki-67 Labeling Index (Ki-67 LI)

Immunohistochemical staining for Ki-67 was employing streptavidin-peroxidase- (SP-) based methods. The primary antibodies and dilutions were used for Ki-67 (MIB-1, 1 : 200, DakoCytomation, Glostrup, Denmark). Paraffin gland blocks were cut into 4-66 *μ*m thick sections and placed on glass slides. Slides were deparaffinized twice in xylene every 20 min and diluted in 100% (10 min), 95% (5 min), 80% (5 min), and 70% (5 min) alcohol degree. Slides were incubated for 10 min in 3% H_2_O_2_ to block endogenous peroxidase, followed by heat-induced antigen retrieval. After incubation in 1% normal horse blood at room temperature for 30 min, the slides were incubated with the primary and secondary reactions. The slides were then dipped in a solution of polymerantibody-peroxidase complex and incubated at room temperature for 30 minutes. Using PBS, the slides were washed 3 times, each for 5 minutes, and reacted in DAB solution and hematoxylin. Finally, the slides were covered with a glass deck and observed by a light microscope. Ki-67-positive cells were counted by averaging 5 visual fields (×200) in each slide.

### 2.5. Statistical Analysis

SPSS 20.0 software was used for statistics. The classification of measurement data is always tested by Shapiro Wilk test. If the data do not fit into the conventional classification, they are presented as a mean (multiple) and analyzed using the Wilcoxon test or the Mann–Whitney *U* test. Correlation between *rD*, *rD*∗, *rf*, *r*CBF, and Ki-67 LI was determined using the Pearson correlation coefficient. The receiver operating characteristic (ROC) and the area under the curve (AUC) were used to measure the diagnosis of *rD*, *rD*∗, *rf*, and *r*CBF in differentiation between advanced and low-level gliomas. If the possibility (*P*) of difference was less than 0.05, the difference was considered statistically significant.

The article "Intravoxel Incoherent Motion Diffusion-Weighted Imaging and 3D-ASL to Assess the Value of Ki-67 Labeling Index and Grade in Glioma" was retracted in 2023. Reasons: signs of a paper mill; compromised peer review; unreliable results or conclusions.

## 3. Results

### 3.1. IVIM-DWI and 3D-ASL Parameters between Tumor and Contralateral Normal White Matter in Patients with Gliomas

The *D*, *D*∗, *f*, and CBF of the tumor solid area were 0.83 (0.52-1.21), 4.46 (1.89-13.44), 0.34 (0.13-0.59), and 81.59 (19.56-225.54), respectively. The *D*, *D*∗, *f*, and CBF of the contralateral normal white matter were 0.65 (0.41-0.95), 3.59 (1.70-20.06), 0.20 (0.09-0.33), and 29.97 (10.56-78.29), respectively. Significant differences were observed between tumor and contralateral normal white matter for IVIM-DWI and 3D-ASL parameters (*P* < 0.05, Table 1, Figures 1 and 2).

### 3.2. IVIM-DWI, 3D-ASL Parameters, and Ki-67 LI between Low-Grade and High-Grade Glioma Patients

Next, we found differences between IVIM-DWI and 3D-ASL in patients with advanced glioma. Grade II glioma patients were included in the low group (*n* = 20), and patients with grades III-IV glioma were included in the high group (*n* = 22). The low-grade group was 52.15 ± 12.36 years, with 9 males and 11 females. The high-grade group was 53.23 ± 12.86 years, with 13 males and 9 females. There was no significant difference between the two age groups and gender distribution. To avoid individual variations among samples, the *D*, *D*∗, *f*, and CBF of the tumor region were relative to those of the contralateral normal white matter for each patient, with *rD*, *rD*∗, *rf*, and *r*CBF obtained. The *rD*, *rD*∗, *rf*, and *r*CBF of low-grade glioma patients were 1.61 (0.88-2.41), 0.99 (0.41-2.64), 2.23 (0.43-4.83), and 1.65 (0.41-9.15), respectively. The *rD*, *rD*∗, *rf*, and *r*CBF of high-grade glioma patients were 1.05 (0.63-1.73), 1.63 (0.33-5.89), 1.29 (0.54-4.27), and 3.49 (0.72-12.17), respectively. Remarkable differences were noted in the *rD*, *rD*∗, *rf*, and *r*CBF between low-grade and high-grade glioma patients (*P* < 0.05, Table 2). The Ki-67 LI of low-grade glioma patients was 0.05 (0.02-0.17) and that of high-grade glioma patients was 0.26 (0.02-0.63), to show the significant differences between the two groups of the patients (*P* < 0.001, Table 2).

### 3.3. Correlation between IVIM-DWI, 3D-ASL Parameters, and Ki-67 LI of Glioma Patients

In this part, we performed Pearson analysis to confirm the correlation between IVIM-DWI, 3D-ASL parameters, and Ki-67 LI of glioma patients, with *r* value ranging 0.71 to 1 as high correlation, 0.41 to 0.70 as moderate correlation, and ≤0.40 as low correlation. Ki-67 LI was found to be negatively correlated with *rD* (*r* = −0.693, *P* < 0.001) and *rf* (*r* = −0.539, *P* < 0.001) but had no correlation with *r*CBF (*r* = 0.665, *P* < 0.001) in glioma patients (Figure 3). However, no significant correlation was noted between *rD*∗ and Ki-67 LI of glioma patients.

The article "Intravoxel Incoherent Motion Diffusion-Weighted Imaging and 3D-ASL to Assess the Value of Ki-67 Labeling Index and Grade in Glioma" was retracted in 2023. Reasons: signs of a paper mill; compromised peer review; unreliable results or conclusions.

### 3.4. Predictive Performance of IVIM-DWI, 3D-ASL Parameters, and Ki-67 LI for Different Grades of Glioma

The *rD*, *rD*∗, *rf*, *r*CBF, and Ki-67 LI of glioma patients were used to predict high-grade glioma patients from low-grade glioma patients. The ROC (as shown in Figure 4) for prediction of high-grade glioma by *rD*, *rf*, *rD*∗, *r*CBF, and Ki-67 LI yielded AUC of 0.819, 0.747, 0.719, 0.836, and 0.907, respectively. The sensitivity and specificity values are presented in Table 3.

## 4. Discussion

Glioma is the most common malignant neoplasm in adults and most commonly occurs in the brain and glial tissues. Currently, there is no unification of the histological classification of glioma, which is often named as similarity of glial cells. According to the WHO 2016 publication, the main gliomas include astrocytoma, oligodendroglioma, a combination of 2 cell types, ependymoma, neuroblastoma, and mixed glioma. Depending on the severity of the cancer, gliomas are classified into I-IV grades [15]. The incidence rate of glioma is 5.26/100,000 each year, and 17,000 cases are diagnosed annually. The patients with glioma are at risk of high mortality, especially for the population with grade IV represented by glioblastoma [16]. Therefore, accurate assessment of glioma level prior to treatment is important in treatment selection and evaluation.

On this study, IVIM and 3D-ASL were applied to the glioma patients with different grades to confirm their diagnostic evaluation. IVIM based on DWI is a contrast agent-free imaging technology, which randomly orients the blood flow of capillaries in tissues to simulate the pseudodiffusion process. It has been considered as an effective method applying to the field of tumor [17]. The approach of ASL is a method for imaging cerebral perfusion and cerebral angiography [18]. The results presented in this study showed that significant difference was found in the median value of *D*, *D*∗, *f*, and CBF between the healthy white matter and tumor solid. Higher median value of *D* in the glioma tissue indicated the diffusion movement of water molecules was remarkably stronger than that in healthy white matter. This might due to the increase of extracellular space caused by the destruction of normal cells. The severity of cancer infiltration was caused by *D*∗, *f*, and CBF indices. Elevations in *D*∗, *f*, and CBF did not directly indicate the presence of numerous microvessels in the glioma tissue [19]. A report by Bisdas et al. found significant differences in *D*, *D*∗, and *f* levels of contralateral health problems white and advanced glioma. These results have been shown to be significantly different in patients with advanced glioma [20]. Togao et al. showed that the value of *D* in the advanced glioma group was lower in the lower group, while the value of *f* in the higher group was lower in the lower group, and there was no difference in *D*∗ values of both groups [21]. These data were a little different from ours, indicating that, comparing to the low-grade group, lower *rf* value and higher value of *rD*∗ were found in the high-grade group. However, our findings above were similar to the report represented by Lin et al. [22]. Chen et al. also showed that the high and low values of *f* on *D*∗ were lower than the higher groups [23]. The differences in the *f* value between the two groups in studies might be related to various factors, such as difference in selected cases, tumor structural characteristics, the selection of *b* value, and setting in parameters of IVIM-DWI. In this study, the *rD* value of the upper group was lower than that of the lower group, which indirectly reflected tumor cells in high-grade glioma had stronger proliferation ability and higher cell density, resulting in limited diffusion of water molecules. Lin et al. demonstrated that higher CBF value was noted in the high-grade glioma, which was similar to our findings.

The article "Intravoxel Incoherent Motion Diffusion-Weighted Imaging and 3D-ASL to Assess the Value of Ki-67 Labeling Index and Grade in Glioma" was retracted in 2023. Reasons: signs of a paper mill; compromised peer review; unreliable results or conclusions.

Ki-67 is a nuclear protein expressed at almost all stages of the cell cycle, and its expression is associated with tumor cell growth. A subset of Ki-67 LI is involved in disease therapy [24]. It was found that the high-grade glioma patients showed significant higher value of Ki-67 LI comparing to the patients with low-grade glioma, indicating the proliferative activity of tumor cells increased with its histological grade, which was proved by other studies [25, 26]. The Pearson analysis in this study revealed that Ki-67 LI expression was negatively correlated with *rD* and *rf*. A similar study indicated the level of *rD* and *rf* in high-grade and low-grade glioma were moderately negatively correlated with the Ki-67 LI [27]. The results indicated the level of *rD* and *rf* was related to changes in proliferative activity and cell density of tumor cells. In addition to this study, no remarkable correlation between *rD*∗ and Ki-67 Li in patients with glioma was discovered, which suggested tumor proliferation activity was not closely associated with blood perfusion. It was found that Ki-67 LI was positively correlated with *r*CBF of glioma patients, indicating the velocity of blood perfusion was related to the tumor proliferation activity. The ROC analysis showed that *rD*, *rf*, *rD*∗, *r*CBF, and Ki-67 LI yielded AUC of 0.819, 0.747, 0.719, 0.836, and 0.907, respectively. The four parameters in IVIM-DWI and 3D-ASL, as well as the fraction of Ki-67 LI, can be used for assessment of grading in human glioma.

The article "Intravoxel Incoherent Motion Diffusion-Weighted Imaging and 3D-ASL to Assess the Value of Ki-67 Labeling Index and Grade in Glioma" was retracted in 2023. Reasons: signs of a paper mill; compromised peer review; unreliable results or conclusions.

In conclusion, the parameters of IVIM-DWI and 3D-ASL are efficient in identifying glioma grade. The present study indicated that the value of *rD*, *rf*, and *r*CBF were closely associated with tumor proliferation activity, which can predict quantitatively the fraction of Ki-67 LI. These parameters contributed to the treatment scheme optimization and prognosis improvement in glioma. However, the data might not be completely reliable due to limited numbers of eligible patients involved in this study. Additionally, the detection of tumor solid area instead of the whole lesion may lead to data deviation. Further studies should be carried out to verify these results.

## Figures and Tables

**Figure 1:** Representative images of the patient with gliomas. The patient was a 66-year-old man who developed a WHO grade II oligodendroglioma in his left frontal lobe.

**Figure 2:** Representative images of the patient with gliomas. The patient was a 57-year-old man who developed a WHO grade III oligodendroglioma in his left frontal lobe.

**Figure 3:** Correlation between *rD*, *rf*, *r*CBF, and Ki-67 LI in glioma patients.

**Figure 4:** Predictive performance of IVIM-DWI, 3D-ASL parameters, and Ki-67 LI for different grades of glioma.

**Table 1:** IVIM-DWI and 3D-ASL parameters between tumor and contralateral normal white matter in patients with gliomas.

ROI	*D*	*D*∗	*f*	CBF
Tumor	0.83 (0.52-1.21)	4.46 (1.89-13.44)	0.34 (0.13-0.59)	81.59 (19.56-225.54)
Contralateral normal white matter	0.65 (0.41-0.95)	3.59 (1.70-20.06)	0.20 (0.09-0.33)	29.97 (10.56-78.29)
*Z*	-3.289	-2.232	-4.180	-4.620
*P*	0.001	0.026	<0.001	<0.001

Statistical analysis was performed using Wilcoxon test.

**Table 2:** IVIM-DWI, 3D-ASL parameters, and Ki-67 LI between low-grade and high-grade glioma patients.

Grade	*rD*	*rD*∗	*rf*	*r*CBF	Ki-67 LI
Low grade	1.61 (0.88-2.41)	0.99 (0.41-2.64)	2.23 (0.43-4.83)	1.65 (0.41-9.15)	0.05 (0.02-0.17)
High grade	1.05 (0.63-1.73)	1.63 (0.33-5.89)	1.29 (0.54-4.27)	3.49 (0.72-12.17)	0.26 (0.02-0.63)
*Z*	-3.540	-2.430	-2.733	-2.166	-4.516
*P*	<0.001	0.015	0.006	0.030	<0.001

Statistical analysis was performed using Mann–Whitney *U* test.

**Table 3:** Predictive performance of IVIM-DWI, 3D-ASL parameters, and Ki-67 LI for different grades of glioma.

	*rD*	*rD*∗	*rf*	*r*CBF	Ki-67
AUC	0.819	0.719	0.747	0.836	0.907
*P*	<0.001	0.015	0.006	<0.001	<0.001
95% CI	0.694-0.945	0.560-0.878	0.589-0.904	0.712-0.961	0.777-1.000
Sensitivity (%)	84.93	73.77	76.23	86.20	90.03
Specificity (%)	83.23	67.58	69.43	85.11	88.84

The article "Intravoxel Incoherent Motion Diffusion-Weighted Imaging and 3D-ASL to Assess the Value of Ki-67 Labeling Index and Grade in Glioma" was retracted in 2023. Reasons: signs of a paper mill; compromised peer review; unreliable results or conclusions.

## Data Availability

The data used to support the findings of this study are included in the sentence.
